This article has been retracted.

# GraphCovidNet: A graph neural network based model for detecting COVID-19 from CT scans and X-rays of chest

**DOI:** 10.1038/s41598-021-87523-1

**Published:** 2021-04-15

**Authors:** Pritam Saha, Debadyuti Mukherjee, Pawan Kumar Singh, Ali Ahmadian, Massimiliano Ferrara, Ram Sarkar

**Affiliations:** 1 Department of Electrical Engineering, Jadavpur University, Kolkata, 700032 India; 2 Department of Computer Science and Engineering, Jadavpur University, Kolkata, 700032 India; 3 Department of Information Technology, Jadavpur University, Kolkata, 700106 India; 4 Institute of IR 4.0, The National University of Malaysia, Bangi, 43600 UKM Selangor Malaysia; 5 School of Mathematical Sciences, College of Science and Technology, Wenzhou-Kean University, Wenzhou, China; 6 ICRIOS-The Invernizzi Centre for Research in Innovation, Organization, Strategy and Entrepreneurship, Department of Management and Technology, Bocconi University, Via Sarfatti, 25, 20136 Milan (MI), Italy

**Keywords:** Viral infection, Computer science

## Abstract

COVID-19, a viral infection originated from Wuhan, China has spread across the world and it has currently affected over 115 million people. Although vaccination process has already started, reaching sufficient availability will take time. Considering the impact of this widespread disease, many research attempts have been made by the computer scientists to screen the COVID-19 from Chest X-Rays (CXRs) or Computed Tomography (CT) scans. To this end, we have proposed **GraphCovidNet**, a Graph Isomorphic Network (GIN) based model which is used to detect COVID-19 from CT-scans and CXRs of the affected patients. Our proposed model only accepts input data in the form of graph as we follow a GIN based architecture. Initially, pre-processing is performed to convert an image data into an undirected graph to consider only the edges instead of the whole image. Our proposed **GraphCovidNet** model is evaluated on four standard datasets: SARS-COV-2 Ct-Scan dataset, COVID-CT dataset, combination of covid-chestxray-dataset, Chest X-Ray Images (Pneumonia) dataset and CMSC-678-ML-Project dataset. The model shows an impressive accuracy of 99% for all the datasets and its prediction capability becomes 100% accurate for the binary classification problem of detecting COVID-19 scans. Source code of this work can be found at GitHub-link.

## Introduction

Recently, Coronavirus (COVID-19) disease has created an unprecedented situation across the world. Severe Acute Respiratory Syndrome coronavirus 2 (SARS-CoV-2), a novel virus enveloped with large single stranded RNA genome^1^ is the root cause for this disease^2^. Although this virus is originated from Wuhan in China, in December 2019, later America and several other countries of Europe have severely affected in early days of the year 2020^3^. According to recent statistics, both America and India have more number of confirmed cases than other affected countries. World Health Organization (WHO)^4^ announced COVID-19 as a global health emergency on January 30, 2020 considering the adverse effects of this situation.

To diagnose the SARS-CoV-2, it has been observed that both CXRs as well as CT-scans are found to be beneficial^5,6^. CXR images are more appreciated by the medical practitioners, since it can be obtained easily from the radiology departments. According to radiologists, CXR images help to understand the chest pathology clearly^1^. However, CT scans provide high sensitivity, for example, 97% of the positive CT scans are confirmed in a case study in Wuhan^7^. Due to the exponential growth in cases, it is required to develop a automated and fast paced system which can identify COVID-19 from chest CT-scans or CXR images. Figure 1 shows some samples of these CT-scan and CXR images.

**Figure 1:** Sample CT scans and CXRs of some patients (source: (i) CT-scan—SARS-COV-2 Ct-Scan Dataset^8^, (ii) CXR—CMSC-678-ML-Project^9^).

SARS-CoV-2 generally affects the lungs and turbid formation of cough around lungs can be detected from CT-scans and CXRs. The usual symptoms of COVID-19 are related to fever, dry cough and tiredness. The severity of COVID-19 symptoms can range from very mild to critical. Some people may show only a few symptoms, and sometimes no symptoms can be observed at all. In some cases, symptoms start worsen mere after a week and frequent shortness of breath and Pneumonia may happen. Elders and people with chronic medical conditions may possess a higher risk of serious illness from COVID-19. Now in case of mild COVID-19, CT-scans and CXR images may be inefficient as the cough clouds may not be prominent. Another failed case for CT-scan and CXR diagnosis may be any other kind of Pneumonia because of the presence of turbid lungs. So, an advanced classification model is needed to classify these CT-scans and CXR properly.

Due to this pandemic, a lot of people have been affected around the world and rapid tests are required with proper treatment and quarantine. Though Real Time Reverse Transcription Polymerase Chain Reaction (RT-PCR) test is the most common way to detect the virus, but the time required to get the results is around 1–2 days^10^. So, an automatic and accurate classification method, where CT-scans or CXRs are used, can be considered as an alternative approach in order to deal with this pandemic whose turn around time is significantly less.

Although spread of COVID-19 has started recently, many research works have already been performed by the researchers during this short time span. Since the current problem consists of classifying COVID-19 images, various machine learning as well as deep learning methods have been proposed. In this section, a few works have been mentioned in brief.

Soares et al.^8^ have used an explainable deep learning model called xDNN on the SARS-CoV-2 CT-scan dataset^8^ and have achieved 97.31% accuracy in the binary classification of scans between COVID and Non-COVID. Yang et al.^11^ have introduced the COVID-CT dataset in their work. Since the total number of images are approximately 700 in the original dataset, they have used segmentation masks for lungs and lesion region to gain additional information from the original images. In their work, Contrastive Self-Supervised Learning (CSSL), an unsupervised learning approach^12^ has been implemented to fine-tune the ImageNet pretrained models DenseNet-169^13^ and ResNet-50^14^. Overall, they have achieved best accuracy as 89.1%. Pedro et al.^15^ have utilized the EfficientNet^16^ model along with transfer learning citetranferlearning and have achieved accuracies 87.60% and 98.99% for COVID-CT dataset^11^ and SARS-CoV-2 CT-scan dataset^8^ respectively. Sharma et al.^17^ have applied ResNet^14^ on the database consisting of datasets: (i) GitHub COVID-CT dataset^11^, (ii) COVID dataset provided by Italian Society of Medical and Interventional Radiology^18^, (iii) dataset provided by hospitals of Moscow, Russia^19^, (iv) dataset provided by SAL Hospital, Ahmedabad, India^20^ and have obtained almost 91% accuracy.

Elaziz et al.^21^ have used a modified version of Manta-Ray Foraging Optimization (MRFO) for feature selection and later have used K-Nearest neighbor (KNN)^22^ for classification. They have considered two COVID datasets: (i) combined database of: covid-chestxray-dataset^23^ and ChestX-Ray Images (Pneumonia) dataset^24^, (ii) dataset provided by Chowdhury et al.^25^. They have achieved 96.09% and 98.09% accuracies on those two datasets respectively. Turkoglu et al.^26^ have proposed an COVIDetectioNet model where they have used transfer learning on a pre-trained Convolutional Neural Network (CNN)^27^ called AlexNet. They have used Relief feature selection algorithm from all the layers of the architecture, and for the classification they have used Support Vector Machine (SVM)^28^. They have conducted their experiments on the combined dataset of: (i) dataset provided by Chowdhury et al.^25^, (ii) Chest X-RayImages (Pneumonia) dataset^24^ and (iii) COVID-19 Radiography Database^29^. Their proposed model has predicted 99.18%. accurate results on the combined dataset. Oh et al.^30^ have performed semantic segmentation by using an extended fully convolutional (FC)-DenseNet103^13^ and later have used ResNet-18^14^ on the combined database of: (i) JSRT dataset^31^, (ii) SCR dataset^32^, (iii) NLM(MC) dataset^33^, (iv) covid-chestxray-dataset^23^, (v) CoronaHack dataset^34^. In their work, 88.9% accurate results have been achieved.

Nour et al.^3^ have proposed a five-layer CNN model on the COVID-19 radiology database^25^. This dataset is composed of different benchmark datasets^18,23,35^. After extracting features from the proposed CNN model, basic machine learning algorithms KNN^22^, SVM^28^ and Decision Tree (DT)^36^ are applied on the extracted features. State-of-the-art result is achieved using SVM with accuracy 98.97%. Chandra et al.^37^ have used majority voting based ensemble of five classifiers—SVM^28^, KNN^22^, DT^36^, Artificial Neural Network (ANN)^38^, Naive Bayes (NB)^39^ on the database consisting of three publicly available CXR image datasets: covid-chestxray dataset^23^, Montgomery dataset^40^, and NIH ChestX-ray14 dataset^41^. Among the total 8196 features extracted from all the pre-processed images, 8 are First Order Statistical Features (FOSF)^42^, 88 are Grey Level Co-occurrence Matrix (GLCM)^43^ based features and the rest 8100 are Histogram of Oriented Gradients (HOG)^44^ features. The proposed classifier ensemble has predicted with 98.06% and 93.41% accuracy for 2 class (normal and abnormal) and 3 class (i.e., normal, COVID-19 and Pneumonia) classification problems respectively.Hemdam et al.^45^ have used seven benchmark image classifier models: VGG19^46^, DenseNet201^47^, InceptionV3^48^, ResNetV2^14^, Inception-ResNet-V2^49^, Xception^50^, MobileNetV2^51^ on the dataset combined from covid-chestxray-dataset^23^ and dataset provided by Dr. Rosebrock^52^. VGG19 and DenseNet201 have provided results with best accuracy as 90%.

Makris et al.^53^ have used various existing CNN models along with transfer learning on the CXR images collected from sources: covid-chestxray dataset^23^ and Chest X-Ray Images dataset by Mooney et al.^24^. Among all the used models, VGG16 and VGG19^46^ have provided the best accuracy as 95%. Zhong et al.^54^ have used a CNN model based on VGG16^46^ architecture on the database consisted of- covid-chestxray-dataset^23^, ChestX-RayImages (Pneumonia) dataset^24^, Figure 1 COVID-19 Chest X-ray Dataset Initiative dataset^55^ and ActualMed COVID-19 Chest X-ray Dataset Initiative dataset^56^. Finally, they have obtained 87.3 % accurate results on their work. Sun et al.^6^ have proposed an Adaptive Feature Selection guided Deep Forest (AFS-DF) algorithm and have achieved 91.79% accurate results on the CT scan database collected from the Third Hospital of Jilin University, Ruijin Hospital of Shanghai Jiao Tong University, Tongji Hospital of Huazhong University of Science and Technology, Shanghai Public Health Clinical Center of Fudan University, Hangzhou First People’s Hospital of Zhejiang University, and Sichuan University West China Hospital.

Chattopadhyay et al.^57^ have contributed in two-ways in their work in this domain. After extracting deep features from the original image dataset, they have applied a completely novel meta-heuristic feature selection approach named Clustering-based Golden Ratio Optimizer (CGRO). They have conducted the necessary experiments on the SARS-COV-2 Ct-Scan Dataset^8^, COVID-CT dataset^11^ and Chest X-Ray dataset^24^ and have achieved the state-of-the-art accuracies of 99.31%, 98.65%, 99.44% respectively.

Sen et al.^58^ have proposed a CNN architecture and bi-stage Feature Selection (FS) approach to extract the most relevant features from the chest CT-scan images. Initially, they have applied a guided FS methodology by employing two filter procedures: (i) Mutual Information (MI), (ii)Relief-F. In the second stage, Dragonfly algorithm (DA) has been used for the further selection of the most relevant features. Finally, SVM has been applied to the overall feature set. The proposed model has been tested on two open-access datasets: SARS-CoV-2^8^ CT images and COVID-CT^11^ datasets and has got 98.39% and 90.0% accuracies on the said datasets respectively.

Besides classification of CT-scans and CXRs, there are other research fields related to COVID-19. One such field is mask detection. Loey et al.^59^ have used first ResNet50^14^ and then an ensemble of DT and SVM for the final classification. They have achieved best results for the SVM classifier with 99.64%, 99.49% and 100% accuracies for the three datasets: e Real-World Masked Face Dataset (RMFD)^60^, the Simulated Masked Face Dataset (SMFD)^61^, and the Labeled Faces in the Wild (LFW)^62^ respectively.

From the above mentioned works, it is clear that in most of the cases pre-existing or novel CNN^27^ models are used as a classifier since this is basically an image classification problem. However, CNN has some limitations, for example, it can be overfitted when there is some class imbalance in the dataset^63^. On the other hand, Graph Neural Network (GNN)^64^ based models can overcome the problems like: overfitting and class imbalance. From the experimental results found in other fields, it is evident that a GNN based model generally works fast^65^. GNN, a relatively new approach in the field of deep learning domain, is applied for graph classification problems. So, GNN requires input data represented in the form of graph data structure. Whereas, any 2D-CNN model directly accepts a 2D image matrix as input. Therefore, we need a proper technique for mapping an image classification problem to a graph classification one. We have resolved this issue with the help of an appropriate pre-processing technique to convert an image into a graph data. Considering all the advantages and novelties of GNN approach, we have implemented our proposed **GraphCovidNet**, a Graph Isomorphism Network (GIN)^66^ based model (a special category of GNN) called **GraphCovidNet**.

The experimental results show that our proposed model performs very well with respect to time-requirement by the model. Our architecture has also performed well for highly class imbalanced dataset due to the injective nature of the aggregation function. The architecture is able to map different graphs into different representations in the embedding space properly. Hence, the proposed model is able to identify the class with a lesser image count perfectly. We have used four publicly available datasets: (i) SARS-COV-2 Ct-Scan Dataset^8^, (ii) COVID-CT dataset^11^, (iii) 3-class and 4-class datasets under CMSC-678-ML-Project^9^, (iv) combination of two datasets: (1) covid-chestxray-dataset available on GitHub^23^, (2) Chest X-Ray Images (Pneumonia) dataset available on Kaggle^24^. The main contributions of our work can be summarized as follows:

- In our work, we have introduced a new classification model, called **GraphCovidNet**, for screening COVID-19 CT-scan and CXR images.
- In the proposed model, we have used GIN as its backbone architecture which falls under a specialized category of GNN. Based on authors’ knowledge, any GNN based architecture has not been used previously in this domain.
- We have mapped image classification problem into a graph classification problem with proper pre-processing technique.
- We have also reduced the space complexity of our model by considering only the edges of an image instead of the whole image which, in turn, makes our approach computationally inexpensive.
- Our approach is not limited to a particular type of input as we have considered both CT-scan and CXR images and we have also worked binary to multi-class classification problem.
- Our model has also surpassed the existing state-of-the-art approaches.

Our proposed method is diagrammatically represented in Fig. 2.

**Figure 2:** Generic framework of our proposed **GraphCovidNet** model for COVID-19 detection from CT-scan or CXR images (Sample CT-scan image source: CT-scan—SARS-COV-2 Ct-Scan Dataset^8^).

Our entire work has several sections that include: (1) Introduction, (2) Results and discussion, (3) Methodology, (4) Conclusion, (5) Data availability and finally, (6) Code availability.

## Results and discussion

In our experiments, we have used 5-fold cross-validation for evaluating the model. During each fold, the training is done for 10 epochs. We have used Adam optimizer and stochastic gradient descent (SGD) approach with a learning rate of 0.001 to train our model.

Here we have used five standard evaluation metrics such as Accuracy, Precision, Recall, F1 Score and Receiver Operating Characteristic (ROC) curve to assess our model performance. Table 1 shows the performance results as well as the average time taken for both training and testing in each fold given by our proposed **GraphCovidNet** model for all the four datasets.

**Table 1:** Detailed results of the proposed **GraphCovidNet** model for all the four datasets in terms of some standard evaluation metrics.

Dataset	Category	Accuracy (%)	Precision (%)	Recall (%)	F1 Score (%)	Training time (s)	Testing time (s)
SARS-COV-2 Ct-Scan Dataset	–	100	100	100	100	342.586	2.328
COVID-CT dataset	–	100	100	100	100	146.365	1.151
covid-chestxray-dataset + Chest X-Ray Images (Pneumonia) dataset	–	99.84	99.84	99.84	99.84	1071.296	7.138
CMSC-678-ML-Project GitHub	3-class	99.11	99.11	99.11	99.11	66.923	0.6
	4-class	99	99	99	99	73.697	0.612

From Table 1, it is clear that the **GraphCovidNet** model has achieved at least 99% accuracy for all the datasets, whereas it gives 100% accuracy for the 2-class datasets. Generally, with increase in number of classes, our proposed model’s prediction capability drops from 100 to 99%. One notable point is that our proposed model provides nearly perfect (99.84%) accuracy for the heavily class imbalanced combined database of- covid-chestxray-dataset, Chest X-Ray Images (Pneumonia) dataset. Intuitively it can be said that a powerful GNN maps two nodes to the same location only if they have identical sub-trees with identical features on the corresponding nodes. Sub-tree structures are defined recursively via node neighborhoods. Thus, we can reduce our analysis to the question whether a GNN maps two neighborhoods (i.e., two multi-sets) to the same embedding or representation. A maximally powerful GNN would never map two different neighborhoods, i.e., multi-sets of feature vectors to the same representation. This means its aggregation scheme must be injective. Thus, it can be said that a powerful GNN’s aggregation scheme is able to represent injective multi-set functions.

### Theorem

Let *A* : $G \rightarrow R^d$ be a GNN. With a sufficient number of GNN layers, *A* maps any graphs, say, *G*1 and *G*2 such that the Weisfeiler–Lehman test of isomorphism decides as non-isomorphic, to different embeddings if the following conditions hold:

- *A* aggregates and updates node features iteratively with $h_v^{(k)} = \phi (h_v^{(k-1)},f({h_u^{(k-1)} : u \in N(v)})$, where the function,*f*, which operates on multi-sets, and $\phi$ are injective.
- $A's$ graph-level readout, which operates on the multi-set of node features, is injective.

The mathematical proof of the above theorem is already reported in^66^. The GIN follows this theorem. As this network is able to map any two different graphs into different embeddings, which helps to solve the challenging graph isomorphism problem. That is, isomorphic graphs are required to be mapped to the same representation, whereas the non-isomorphic ones to different representations. Due to these reasons, the proposed model even works well on heavily class imbalanced datasets. Based on the data from Table 1, it is also notable that our proposed model takes considerably less time both in training (1–18 min) and testing (0.6–7 s) phases. Less number of epochs is also responsible for such low training time. But again, training loss becomes very less from the very beginning. So, there is no need to consider a large number of epochs for training purpose. We can visualize this low training loss from Fig. 3.

**Figure 3:** Graphical representation of training loss and training accuracy vs epoch for each of the chosen datasets.

In Fig. 3, it is evident that at the first epoch, accuracy is at least 99%, whereas the loss is barely 0.4 for each of the datasets. Further, training reduces the loss value to almost 0, whereas the classification accuracy remains either almost the same or slightly increases with increasing epoch size. Since the change in loss is more prominent as compared to the change in overall accuracy, however, the accuracy seems constant as seen from Fig. 3. Due to proper pre-processing, the proposed architecture is able to understand the input graphs properly. Thus the loss becomes very low from beginning and training gets completed in at most 10 epochs. To verify more about the goodness of our classification model, we have generated Receiver Operating Characteristic (ROC) curves for each of the datasets which are shown in Fig. 4. Additionally, we have conducted experiments by varying the training to testing ratio from 10% to 90% with an interval of 10%. To have a better visualization, we have generated graphs of training and testing accuracies vs training to testing ratio for each of the datasets which are shown in Fig. 5.

**Figure 4:** ROC curves generated by our proposed **GraphCovidNet** model for each of the datasets.

**Figure 5:** Graphical representation of training and testing accuracies vs training ratio for each of the chosen datasets.

So, from Fig. 4, it is evident that for all kind of training to testing ratios, the **GraphCovidNet** model predicts at least 95% samples correctly, which is a sign of its robustness. Figure 5 further proves its success as a classifier because the Area Under the Curve (AUC) for each of the ROC curves is 0.97 units at worst. the AUC for both 2-class datasets is 1 unit and ROC is also perfect. In short, the **GraphCovidNet** model is able to deal with both of the 2-class datasets regardless of the training to testing ratio. We have also conducted experiments on different datasets having equal number of classes for both training and testing purposes. The results of all such training-testing combinations are enlisted in Table 2.

**Table 2:** Detailed results of the proposed **GraphCovidNet** model for all combination of different train-test datasets having same number of classes.

Train data	Test data	Number of classes	Accuracy (%)	Precision (%)	Recall (%)	F1 Score (%)
SARS-COV-2 Ct-Scan Dataset	COVID-CT dataset	2	100	100	100	100
COVID-CT dataset	SARS-COV-2 Ct-Scan Dataset	2	100	100	100	100
covid-chestxray-dataset + Chest X-Ray Images (Pneumonia) dataset	CMSC-678-ML-Project GitHub (3-class)	3	98.78	99.02	97.98	98.54
CMSC-678-ML-Project GitHub (3-class)	covid-chestxray-dataset + Chest X-Ray Images (Pneumonia) dataset	3	99.32	99.23	99.45	99.30

Table 2 shows that proposed model ensures accuracy above 98% even when training and testing data are from two different sources. Such highly accurate results further confirm the validity of **GraphCovidNet**.

To further ensure the superiority of our proposed model, we have also compared its performance against some pretrained CNN models such as Inception-ResNet-V2^49^, VGG19^46^, ResNet152^14^, DenseNet201^47^, Xception^50^, MobileNetV2^51^ for both raw and edge-mapped images. Table 3 shows the accuracies (%) obtained in all the experiments considering the mentioned CNN models.

**Table 3:** Accuracies(%) obtained by applying Inception-ResNet-V2, VGG19, ResNet152, DenseNet201, Xception, MobileNetV2 models for both raw and edge-mapped images.

Model	SARS-COV-2 Ct-Scan Dataset		COVID-CT dataset		covid-chestxray-dataset + Chest X-Ray Images (Pneumonia) dataset		CMSC-678-ML-Project GitHub (3-class)		CMSC-678-ML-Project GitHub (4-class)	
	Raw image	Edge image	Raw image	Edge image	Raw image	Edge image	Raw image	Edge image	Raw image	Edge image
Inception-ResNet-V2	77.85	80.08	74.35	78.95	98.22	98.05	82.61	91.3	77.56	86.45
VGG19	78.27	82.55	79.60	84.27	98.45	96.50	86.96	97.83	79.65	92.2
ResNet152	77.87	84.58	86.65	87.97	98.68	97.82	91.31	91.40	86.13	85.88
DenseNet201	75.86	85.69	89.11	90.21	99.07	97.35	95.65	96.13	88.65	90.44
Xception	83.30	81.79	82.01	87.58	96.74	99.22	82.61	86.96	82.15	83.97
MobileNetV2	77.46	80.48	78.18	76.97	98.76	98.52	93.48	84.74	81.45	82.25

Comparison between Tables 1 and 3 validates that **GraphCovidNet** outperforms all these conventional CNN models which gives a more clear view about the robustness of our proposed model.

We have also compared the results of our proposed **GraphCovidNet** model with some past works done on the chosen datasets. Table 4 demonstrates such comparative results.

**Table 4:** Comparison of our proposed **GraphCovidNet** model with some previous works on all the datasets (Oh et al.^30^, Chandra et al.^37^, Nour et al.^3^, Hemdam et al.^45^, Turkoglu et al.^26^ have combined other dataset; Oh et al.^30^, Chandra et al.^37^, Hemdam et al.^45^ have considered the first dataset only; Nour et al.^3^, Turkoglu et al.^26^ have considered the second dataset only).

Dataset	Authors	Methodology	Accuracy (%)	Precision (%)	Recall (%)	F1-score (%)
SARS-COV-2 Ct-Scan Dataset^8^	Soares et al.^8^	xDNN	97.38	99.16	95.53	97.31
	Pedro et al.^15^	EfficientNet with transfer learning	98.99	99.20	98.80	99
	Proposed	GraphCovidNet	100	100	100	100
COVID-CT dataset^11^	Pedro et al.^15^	EfficientNet with transfer learning	87.68	93.98	79.59	86.19
	Yang et al.^11^	Segmentation masks with CSSL	89.1	–	–	89.6
	Proposed	GraphCovidNet	100	100	100	100
covid-chestxray-dataset^23^+Chest X-Ray Images (Pneumonia) dataset^24^	Makris et al.^53^	VGG16 and VGG19 with transfer learning	95.88	COVID-96 normal-95 Pneumonia-95	COVID-96 normal-100 Pneumonia-91	COVID-98 normal-98 Pneumonia-98
	Elaziz et al.^21^	MRFO + KNN	96.09	98.75	98.75	98.75
	Zhong et al.^54^	VGG16 based CNN model	87.3	89.67	84.4	86.96
	Oh et al.^30^	DenseNet103 for segmentation + ResNet-18	88.9	83.4	85.9	84.4
	Chandra et al.^37^	Majority voting of SVM, KNN, DT, ANN, NB	93.41	–	–	–
	Nour et al.^3^	CNN for feature extraction + SVM	98.97	–	89.39	96.72 (F-score)
	Hemdam et al.^45^	VGG19 or DenseNet201	90	COVID-83 Normal-100	COVID-100 Normal-80	COVID-91 Normal-89
	Turkoglu et al.^26^	AlexNet+ Relief feature selection algorithm and SVM	99.18	99.48	99.13	99.30
	Proposed	GraphCovidNet	99.84	99.84	99.84	99.84

From Table 4, it is clear that our proposed approach surpasses all the previous works considered here for comparison in terms of accuracy. Although some of the listed previous works are done on database different or even larger than ours, the **GraphCovidNet** model still outperforms the ones on the same dataset. Based on our knowledge, there are no previous works performed on the CMSC-678-ML-Project GitHub dataset^9^. Still there are very few works previously done on a 4-class database in the domain of COVID-19 classification. So, we have considered to note down the results of CMSC-678-ML-Project GitHub dataset^9^. Not only that, any deep learning network generally is unable to achieve high accuracy for very less number of input samples such as CMSC-678-ML-Project GitHub dataset^9^. But **GraphCovidNet** is able to predict with 99% and 99.11% accuracy for its 3-class and 4-class cases respectively as shown in Table 1. So, our proposed model is able to perform very well even in case of datasets having very small number of samples.

In a nutshell, we can say that our proposed model is very accurate, and robust with respect to other existing models.

## Methodology

In this section, we have discussed our proposed work along with the proper pre-processing required for COVID-19 image classification. We have also described the benchmark datasets briefly. This section consists of three subsections: (i) Datasets used, (ii) Pre-processing, and (iii) Proposed model.

### Datasets used

In our work, we have selected the following four datasets to conduct the experiments individually-

1. SARS-COV-2 Ct-Scan Dataset^8^, a 2-class CT scan dataset collected by Plamen et al. available on Kaggle.
2. COVID-CT dataset^11^, a 2-class CT scan dataset introduced by Yang et al. available on GitHub.
3. 3-class dataset which is consisted of CXR from the two sources-
  covid-chestxray-dataset^23^ collected by Cohen et al. available on GitHub.
  Chest X-Ray Images (Pneumonia) dataset^24^ collected by Mooney et al. available on Kaggle.
  For combining these two datasets, we have considered COVID-19 patients’ scans from the covid-chestxray-dataset and normal, Pneumonia patients’ scans from the Chest X-Ray Images (Pneumonia) dataset.
4. Finally, 3-class and 4-class CXR datasets under the CMSC-678-ML-Project available on GitHub^9^

In this section, at first we look at the datasets used in the present work than training constraints alongside the detailed results of the experiments.

Basically, all the 2-class datasets contain classes of COVID and Non-COVID whereas the 3-class datasets contain: Normal, COVID, and Pneumonia. For the 4-class dataset of CMSC-678-ML Project, there are two separate classes of Pneumonia, which are: Bacterial Pneumonia and Viral Pneumonia. Table 5 illustrates the details of these datasets.

**Table 5:** Statistical description of all the datasets used for experimentation.

Dataset	Number of classes	Scan-type	Total number of images		
			Normal	COVID-19	Pneumonia
SARS-COV-2 Ct-Scan Dataset^8^	2	CT	1229	1252	–
COVID-CT dataset^11^	2	CT	407	349	–
covid-chestxray-dataset^23^+Chest X-Ray Images (Pneumonia) dataset^24^	3	CXR	1592	504	4343
CMSC-678-ML-Project GitHub dataset^9^	3	CXR	79	69	79
	4	CXR	79	69	Bacterial: 79, Viral: 79

### Pre-processing

As mentioned earlier, the CT scans or CXRs are first pre-processed in order to apply our proposed **GraphCovidNet** model. We have considered two stages for pre-processing, which are illustrated as follows:

1. Edge detection: First, the edges of the raw images are estimated using Prewitt filter^67^.
2. Graph preparation: Next, these edge maps are converted into graph dataset by proper means.

Now these two stages are explained to have a better understanding of the whole pre-processing part.

#### Edge detection

Basically, an edge is a region denoting a local change of intensity in an image which means that a local maxima or minima will occur for the change of intensity in the edge region. By applying proper filter on the original image, the edges can be prominent. In our work, we have convoluted the original image matrix with 3*3 Prewitt filter^67^ for both horizontal and vertical edge detection which are defined as: $$\begin{bmatrix} -1 &{}&{} -1 &{}&{} -1\\ 0 &{}&{} 0 &{}&{} 0\\ 1 &{}&{} 1 &{}&{} 1\\ \end{bmatrix}$$ and $$\begin{bmatrix} -1 &{}&{} 0 &{}&{} 1\\ -1 &{}&{} 0 &{}&{} 1\\ -1 &{}&{} 0 &{}&{} 1\\ \end{bmatrix}$$ respectively. We have selected Prewitt operator for this experiment because it is easy to implement and it detects the edges quite efficiently^68^. Comparison among the three most popular edge filters: Canny, Sobel and Prewitt applied on a COVID-CT image is shown in Fig. 6. Figure 6 reveals that Sobel filter is the most noisy one, whereas Canny filter produces the least noisy image. Although image produced by Prewitt filter is more noisy than Canny, all edges have different pixel intensity in the case of Prewitt unlike Canny. So choosing pixel value as feature would be wiser for Prewitt filter.

**Figure 6:** Comparison between original COVID-CT image and edge image after applying—Prewitt, Canny and Sobel filters respectively (raw image source: COVID-CT dataset^11^).

After applying convolution on each 3 $\times$ 3 sub-matrix by both of the horizontal and vertical filters, gradient for each sub-matrix has been evaluated. Since all the images are in grayscale, we have considered that a pixel would be situated in an edge if the magnitude of the gradient crosses halfway i.e., the gradient value is greater than or equal to 128. We can get a more clear view of the edge-detection step from Fig. 7.

**Figure 7:** Diagram representing flow of edge-detection method (raw image source: CT-scan—SARS-COV-2 Ct-Scan Dataset^8^).

#### Graph preparation

After the Prewitt filter^67^ is applied on an image, each image is converted to graph. The graph preparation is done using a 3-step procedure which is discussed below:

1. Each pixel having grayscale intensity value greater than or equal to 128 is qualified as a node or a graph vertex. This implies that nodes reside only on the prominent edges of the edge image. Feature of a node consists of the grayscale intensity of the corresponding pixel.
2. Edge exists between the two nodes which represent neighboring pixels in the original image.
3. For each image, one graph is formed. This means that all the nodes as well as the edges constructed from a single image belongs to the same graph. The node attributes, which are simply grayscale values, are normalized graph-wise. Finally, normalization is done by subtracting the mean of all attributes under a graph from the original value and then dividing it by the standard deviation.

Since nodes are formed only from edges present in an image instead of the whole image, so less memory is consumed to prepare such data. Since COVID-19 and any kind of Pneumonia scans contain cloudy region for coughs, detected edges would be different as well as the nature of the graph. This difference might be useful later for classification. Overall five kind of datasets are formed to represent the graph data of all the scans, which are-

1. Node-attribute-dataset: Here the attribute value (in this case the normalized grayscale value) of each node is stored.
2. Graph-indicator-dataset: Here the graph-id for each node is stored.
3. Node-label-dataset: Here the class-label for each node is stored. Since this is a graph level classification, each node under same graph would have same label which is actually the class-label for the corresponding graph.
4. Graph-label-dataset: Here the class-label for each graph is stored.
5. Adjacency-dataset: Here the adjacency sparse matrix for all the graphs is stored.
  Figure 8 summarizes the whole edge-preparation process.

**Figure 8:** Diagram representing the flow of edge-preparation stage.

### Proposed model

We have introduced our novel approach named as **GraphCovidNet**, where we have implemented GIN for classification and prediction tasks. So, before we move deeper into the architecture we will briefly discuss about the graphs, GNN and GIN.

#### Graph neural network

A graph *g* can be described by set of components, nodes (*V*) and edges (*E*) as $g=(V,E)$, where *V* is the set of vertices and *E* is the set of edges. The GNN can be used to classify an unlabelled node in a graph, where some nodes in the graph are labeled using a supervised learning technique. Also, it can do graph classification tasks where each graph has its corresponding labels. Now here, we have formed one graph from each labelled image and have used supervised learning to classify these graphs.

#### Embeddings and graph isomorphism network

In GNN, the nodes of a graph are embedded into a *d*-dimensional embedded space denoted as $h_v$. These nodes are encoded in such a way that the connected nodes or the nodes which have same neighbors are close to each other in embedded space and vice versa. Every node uses its own feature vector $f_v$ and its neighborhood embedding vector $h_{nev}$ to find out it own embedding vector $h_v$.

GNNs uses the graph structure and node features to learn a representation vector of a node, $f_v$, where each node contains the feature vectors, $f_v$ $\forall$ v $\in$ V and each edge contains the feature vectors, $f_e$, $\forall$ e $\in$ E or the entire graph, $h_g$, where $h_g$ = $Readout({h_v, \forall v \in V})$ , where $h_v$ is the final embeddings of the node V is set of all nodes in the graph g. Now every node defines a computation graph based on its neighborhood i.e., every node has its own neural network architecture^64^. This is shown in Fig. 9.

**Figure 9:** Diagram representing the computation graph of a node in an arbitrary graph.

The model for each node can be of arbitrary length. GNN follows a neighborhood aggregation strategy, where we iteratively update the representation of a node by aggregating representations of its neighbors. Nodes have embeddings at each layer. First layer of node is the input feature of that node and after k iterations of aggregation, a node’s representation captures the structural information within its k-hop network neighborhood. Let $x_v$ be the feature vector of the node and $h_{v}^{0}$ be the initial layer embedding. Now, $h_{v}^{0}$ = $x_v$, initial layer embeddings are equal to feature vectors. Formally, the k-th layer of a GNN is

$a_v^{k} = Aggregate^{(k)}({h_u^{(k-1)} : u \in N(v)}) , Combine^{(k)}(h_v^{(k-1)},a_v^{k})$ where, $h_v^{(k)}$ is the feature vector of node v at the k-th layer and $ha_v^{(k)}$ is the aggregated message from its neighborhoods. *N*(*v*) is a set of nodes adjacent to *v*. The choice of $Aggregate^{(k)}$ ($\cdot$) and $Combine^{(k)}$ ($\cdot$) in GNNs are crucial.

Different architectures for *Aggregate* function have been proposed. In the pooling variant of GraphSAGE^69^, *Aggregate* has been calculated as $a_v^{k} = Max({ReLU(b^{(k)} * h_u^{(k-1)}) : u \in N(v)})$ where $b^{(k)}$ is a parameter metrics, and Max represents an element-wise max-pooling. The *Combine* step could be a concatenation of its neighborhood aggregation and its previous layer’s embedding$\cdot$ $h_v^{(k)} = w^{(k)} * Concat(h_v^{(k)},a_v^{k})$ as in GraphSAGE, here $w^{(k)}$ is a parameter metrics. In Graph Convolutional Networks (GCN)^70^, the element-wise mean pooling is used instead, and the *Aggregate* and *Combine* steps are integrated as follows: $h_v^{(k)} = ReLU(W^{(k)} * mean({h_u^{(k-1)}), \forall u \in N(v) })$ .

Mean and max-pooling aggregators are still well-defined multi-set (contains the feature vectors of adjacent nodes of a particular node) functions because they are permutation invariant. But, they are not injective. When performing neighborhood aggregation, the mean(GCN) or max(GraphSage) pooling always obtains the same node representation everywhere. Thus, in this case mean and max pooling aggregators fail to capture any structural information of the graph^66^. GNNs and the Weisfeiler–Lehman (WL) graph isomorphism test^71^, a powerful test known to distinguish a broad class of graphs^72^, are very closely connected.

The WL test has aggregated the labels of nodes and their neighborhoods iteratively and then it hashed the aggregated labels into unique new labels. The algorithm decides that two graphs are non-isomorphic if at some iteration the labels of the nodes between the two graphs differ.Each iteration of WL test has been described as follows: FOR ALL vertices v $\in$ g

1. Compute a hash of $(h_v,h_{v_1},\ldots ,h_{v_n})$ where $h_{v_i}$ are the attributes of the neighbors of vertex v.
2. Use the computed hash as vertex attribute for v in the next iteration.

The algorithm will terminate when this iteration has converged in terms of unique assignments of hashes to vertices.

The WL test is so powerful due to its injective aggregation update that maps different node neighborhoods to different feature vectors. Our key insight is that a GNN can have as large distinguishable power as the WL test if the GNN’s aggregation scheme is highly expressive and can model injective functions. This task to map any two different graphs to different embedding have implied solving graph isomorphism problem. That is, we want isomorphic graphs to be mapped to the same representation and non-isomorphic ones to different representations. Now, the GIN that satisfies the conditions for WL test and generalizes it and hence achieves maximum discriminative power among GNNs. The k-th layer embedding of GIN is given by: $h_v^{(k)} = MLP^{(k)}((1+\epsilon ^{(k)}) * h_v^{(k)} + \sum _{u \in N(v)} h_u^{(k-1)})$, where MLP stands for Multi Layer Perception and $\epsilon ^{(k)}$ is a floating point value.

Now for node classification, the node representation $h_v^{(k)}$ of the kth layer is used for prediction. For graph classification, the *Readout* function aggregates node features from the final iteration to obtain the entire graph’s embedding $h_g$ that is given by the following equation :

$h_g = Readout({h_v^{(k}, \forall v \in V})$. After we have got the embedding of the final layer, a supervised learning for node or graph classification (in our case) needs to be performed.

#### Architecture of our proposed **GraphCovidNet** model

Our architecture consists of a block of GINConv layer which uses MLP^66^ in its subsequent layers for the neighborhood aggregation. In MLP, we have used a block of sequential layers which consist of a linear layer, then a Rectangular Linear Unit (ReLU) layer, followed by another linear layer. It is shown in Fig. 10.

GINConv layer basically takes two different inputs:

1. *x* which is the feature matrix of each node with dimension v*d, where *V* is the total number of nodes in the graph and *d* is embedded dimension.
2. The edge index *E* has a dimension of 2*L consisting of all edges present in the entire graph in the form of pair (*v*1, *v*2), where *v*1 and *v*2 are two nodes connected by an edge and L is the total number of edges in the entire graph.

The output of the GINConv layer is passed through ReLU activation function to introduce non-linearity and then we apply a dropout of 0.5 and it is followed by a normalization (*norm*) layer, which applies layer normalization over a mini-batch of inputs. This output (*out*1) is passed on to another block of the same GINConv-ReLU-dropout-norm layers whose output is *out*2. Now, this *out*2 is passed onto a block which consists of GINConv-ReLU-dropout layers and then it is followed by a global mean pooling layer. After that, a linear layer followed by a dropout layer with dropout rate is equal to 0.5, and then a linear layer with dimension is equal to that of the number of classes of the problem under consideration. Finally, we have used a Log Softmax as the activation function that is used to produce the final probability vector, *z*. The whole architecture is shown in Fig. 11

1 $$\begin{aligned} logsoftmax(z_i) = \log \left( \frac{e^{z_i}}{\sum _{j=1}^{c} e^{z_j}}\right) \end{aligned}$$

where, $z_i$ is the probability of the *ith* element in the last linear layer vector and $\sum _{j=1}^{c} e^{z_j}$ is the sum of all probability values of all the elements including in the vector for the number of classes. We have used negative log likelihood (*nll*) function as the objective function for classification which needs to be minimized and can be represented as follows: *nll*(*z*) $=$ − $\sum _{i=1}^{c} (y_i * logsoftmax(z_i))$ where, $y_i$ is the ground truth label of the ith graph.

**Figure 10:** Diagram representing the MLP architecture of GINConv Layer.

**Figure 11:** Overall architecture of our proposed **GraphCovidNet** model.

## Conclusion

For the past one year, COVID-19 has affected our social and economical lives greatly. In this situation, researchers are focusing on CT scan and CXR images for screening COVID-19 cases of the affected persons. In this paper, we have proposed a novel model, named as **GraphCovidNet**, which basically deals with classification of COVID-19 or any kind of Pneumonia patients from healthy people. Prewitt filter^67^ has been used in the pre-processing stage which produces the edges of an image. Thus our proposed approach utilizes the memory more optimally than the typical CNN based models. Proposed model performs impressively well over different dataset considered in the present work. For some cases, its prediction accuracy even reaches to 100% and it can easily overcome the problems like overfitting and class imbalance. The proposed model has also outperformed many past models in terms of accuracy, precision, recall and f1-score. In future, we can apply the proposed **GraphCovidNet** in other COVID-19 or other medical datasets having CT-scans or CXRs. To be precise, GNN based models are applicable in any kind of image classification problems. We have conducted the present experiments using only 10 epochs to build the training model. So in future, we shall try to improve our model’s speed so that it can be trained in very less time even for larger number of samples.

## Data Availability

No datasets are generated during the current study. The datasets analyzed during this work are made publicly available in this published article.

## Code availability

The codes used for this research work are made publicly available in the GitHub repository: https://github.com/debadyuti23/GraphCovidNet.
